# A descriptive study of a manual therapy intervention within a randomised controlled trial for hamstring and lower limb injury prevention

This article has been retracted.

**DOI:** 10.1186/1746-1340-18-23

**Published:** 2010-08-09

**Authors:** Wayne Hoskins, Henry Pollard

**Affiliations:** 1 Department of Chiropractic, Faculty of Science, Macquarie University, NSW 2109, Australia

## Abstract

**Background:**

There is little literature describing the use of manual therapy performed on athletes. It was our purpose to document the usage of a sports chiropractic manual therapy intervention within a RCT by identifying the type, amount, frequency, location and reason for treatment provided. This information is useful for the uptake of the intervention into clinical settings and to allow clinicians to better understand a role that sports chiropractors offer.

**Methods:**

All treatment rendered to 29 semi-elite Australian Rules footballers in the sports chiropractic intervention group of an 8 month RCT investigating hamstring and lower-limb injury prevention was recorded. Treatment was pragmatically and individually determined and could consist of high-velocity, low-amplitude (HVLA) manipulation, mobilization and/or supporting soft tissue therapies. Descriptive statistics recorded the treatment rendered for symptomatic or asymptomatic benefit, delivered to joint or soft tissue structures and categorized into body regions. For the joint therapy, it was recorded whether treatment consisted of HVLA manipulation, HVLA manipulation and mobilization, or mobilization only. Breakdown of the HVLA technique was performed.

**Results:**

A total of 487 treatments were provided (mean 16.8 consultations/player) with 64% of treatment for asymptomatic benefit (73% joint therapies, 57% soft tissue therapies). Treatment was delivered to approximately 4 soft tissue and 4 joint regions each consultation. The most common asymptomatic regions treated with joint therapies were thoracic (22%), knee (20%), hip (19%), sacroiliac joint (13%) and lumbar (11%). For soft tissue therapies it was gluteal (22%), hip flexor (14%), knee (12%) and lumbar (11%). The most common symptomatic regions treated with joint therapies were lumbar (25%), thoracic (15%) and hip (14%). For soft tissue therapies it was gluteal (22%), lumbar (15%) and posterior thigh (8%). Of the joint therapy, 56% was HVLA manipulation only, 36% high-HVLA and mobilization and 9% mobilization only. Of the HVLA manipulation, 63% was manually performed and 37% mechanically assisted.

**Conclusions:**

The intervention applied was multimodal and multi-regional. Most treatment was for asymptomatic benefit, particularly for joint based therapies, which consisted largely of HVLA manipulation techniques. Most treatment was applied to non-local hamstring structures, in particular the knee, hip, pelvis and spine.

## Background

Hamstring injuries are the most common muscle injury in running based power sports [1]. In Australian Rules football, hamstring injuries are the most prevalent injury, resulting in more missed competition match play than any other injury, whilst other lower-limb muscle strains also feature prominently [2]. The prevention of hamstring and lower limb muscle strains has remained an enigma to the sports clinician. Traditionally, hamstring prevention has focused on local hamstring factors and included warm up, muscle strength and balance, flexibility and fatigue [3]. Orchard has stated that sports medicine dogma counsels that these factors are important in injury prevention, although the scientific evidence for this is sadly lacking [4]. A lack of variety and progression in various prevention and management strategies has been discussed [5], which may be contributing to hamstring injuries remaining a perpetual cause of frustration for athletes and sports clinicians alike.

Whilst the application of manual therapies in the management of hamstring and other sporting injuries has been applied for some time [6,7], its use has remained scarce in more recent scientific literature and research. If used in clinical practice for hamstring injury management, manual therapies typically involve massage and slow velocity spinal mobilizations or slump stretching [8]. Much has been said recently about the role of non-local factors in hamstring injury risk [9,10], and the potential benefits of high velocity spinal and extremity joint manipulation in hamstring injury management [1,5,11]. This has included calls for research incorporating manipulation directed at local and non-local to hamstring areas [5,11]. In addition, despite hands-on therapies being universally used clinically in prevention efforts of sporting injuries, documentation of the various approaches used in the scientific literature is almost non-existent.

There is much controversy [12,13] and little literature describing the use of chiropractic manipulative therapy performed on athletes [14,15]. In particular there is a lack of clinical surveys documenting sports chiropractic treatment techniques and scope of practice. A requirement exists for clinicians of all professions falling under the sports medicine banner to document their clinical practice, as others have done [16-19]. As is the case in the low back pain literature [20], the use of management approaches in sports medicine clinical trials should be documented, particularly if beneficial results are reported. This will assist manual therapists to evolve their management strategies by making treatment decisions based upon the results of clinical trials, allow reproducibility of the study and to allow clinicians to better understand the role that other professions offer to assist in the multidisciplinary management of athletes in an athlete centered approach.

Therefore, we performed a descriptive analysis of the usage of a sports chiropractic manual therapy intervention within a recent randomised controlled trial of semi-elite Australian Rules football players [21]. The study compared the addition of the intervention to the current best practice medical, paramedical and sports science management. It resulted in the significant prevention of lower-limb muscle strains (p = 0.025) with a non-statistically significant trend towards hamstring strains (p = 0.051) and non-contact knee injuries (p = 0.051) [21]. Reductions in overall (p = 0.006) and current low back pain (p = 0.026) were also achieved. A Cochrane systematic review of the literature reviewed the studies methodology and stated that the study exhibited strong external validity [22], whilst a self rated assessment of the trials internal validity using the PEDro criteria rated the study as 'good' [23]. Another strength of the study is the 'missed match' injury definition, which is the only injury definition with proven reliability [24]. The weakness of the study is that it failed to achieve the numbers as determined by the power analysis due to the late withdrawal of two clubs who had previously committed to participation in the study, meaning there is a strong likelihood of a type 2 error in the results [21]. It was the aim of this manuscript to document the type of treatment delivered, whether joint based or soft tissue based, the amount of treatment, the frequency of treatment, to what regions of the body it was directed and to perform a breakdown of the treatment provided into that for symptomatic benefit and that for asymptomatic benefit. Whilst clinical decision making with respect to diagnostic and treatment decisions in the health sciences are often based on previous training, experience and are often considered an art form, publishing of the treatment rendered in this trial is an attempt to allow clinicians to base management decisions upon the results of clinical trials, such that a more scientific component is incorporated into injury management. In particular this information may promote the uptake of newer, non-traditional approaches to injury prevention and management, which may assist in the reduction of hamstring and other lower-limb injuries on a larger scale [25]. Additionally, the publication of these findings may lead to greater awareness of professional roles associated with inter-professional acceptance and optimal standards of care [26].

## Methods

### Participation and randomization

Full details of participation and randomisation have been published elsewhere [21].

Players were eligible to participate if they were listed players on their respective Victorian Football League (VFL) squad and did not meet the exclusion criteria [21]. Fifty-nine players drawn from two of the thirteen clubs competing in the semi-elite state based (VFL) met the studies entry requirements and were randomised into the intervention (n = 29) or control group (n = 30). The clubs, coaches and medical staff gave permission to participate in the trial. Subjects completed informed consent forms to participate and were informed about the purpose and procedures of the study. The procedures used in this study were in accordance with the ethical standards of the Committee on Human Experimentation of Macquarie University (Ethics Approval Number: HE27AUG2004-RO3066).

### Intervention

During the 8 month study, all players from the intervention and control group both continued to receive what can be considered the current best practice management including medication, surgery, manipulative physiotherapy, massage, strength and conditioning and rehabilitation as directed by club staff. All treatment and management from medical, paramedical and sports science staff was independently administered without restriction or interference from the study authors. All medical staff which comprised of at a minimum: doctors, physiotherapists, strength and conditioning staff, trainers and massage therapists were employed by the club and had no limitation in the number of treatments or the type of treatment they could render. The intervention group additionally received a sports chiropractic intervention delivered by a single sports chiropractor (WH). The intervention was pragmatically and individually determined and could involve high velocity, low amplitude (HVLA) manipulation (either manual or mechanically assisted techniques), mobilization (see Table 1[27]) and/or soft tissue therapies: various stretching and soft tissue massage techniques to the spine, pelvis and extremity. Treatment scheduling was also pragmatically and individually determined. During the first 6 weeks of the study players were required to receive one treatment per week minimum. For the next 3 months of the study players were to receive one treatment per fortnight minimum and for the final 3 months of the season (until the completion of the finals series) players were to receive one treatment per month minimum. The study commenced during the pre-season period, 6 weeks prior to round 1 of the regular home and away season.

**Table 1:** Manual therapy definitions

Manipulation	A brief, shallow, sudden carefully administered thrust (high velocity in nature)
Mechanically assisted manipulation	Manipulation performed through the assistance of devices (drop tables or portable drop piece units) or instruments (Activator instruments) being non-cavitational but high velocity in intent

Mobilisation	When a joint is passively moved within its normal range of motion (usually a slow oscillatory movement)

### Data collection

Treatment for the 29 players in the intervention group (mean age 20.2, SD 1.8, range 18-27) for the entirety of the study was continuously recorded by the treating sports chiropractor. Treatment was determined as either being for the purpose of symptomatic benefit for an athlete-reported symptomatic complaint or for asymptomatic functional improvement. Treatment was further broken down as either being joint based (manual or mechanically assisted HVLA manipulation or mobilization) or soft tissue based (soft tissue massage techniques or stretching techniques) and categorized into the various regions of the body to which it was applied (see Table 2). Extremity joints and extremity soft tissue regions were classified as being separate (i.e.: left and right), while spine based treatment was considered as being one on the basis that the effects of manipulation are not limited to a single spinal joint. If multiple treatments were delivered to the same region on the same consultation (e.g. more than one manipulative technique or massage and stretching technique) then this was only recorded once. An analysis of the joint based treatment was conducted to determine the amount of HVLA manipulation only, HVLA manipulation and mobilization, or mobilization only rendered to each joint based region. For the total HVLA manipulation performed, a breakdown was performed to determine the type of technique used, either being manually performed or mechanically assisted.

**Table 2:** The regions/joints managed with joint based therapy

Region	Definition
Foot	All joints distal to the talocrural joint

Ankle	The talocalcaneal, talonavicular, talo-crural and distal tibial-fibular joints

Knee	The patellar-femoral articulation, tibial-femoral articulation and the proximal tibial-fibular joint

Hip	The femoral-acetabular articulation

Sacroiliac joint	The sacroiliac articulation

Pubic symphysis	The public symphysis

Lumbar	The articulation of the 5 lumbar vertebrae and lumbo-sacral joint

Thoracic	The articulation of the 12 thoracic vertebrae

Cervical	The articulation of the 7 cervical vertebrae and the skull

TMJ	The temporomandibular joint articulations

Ribs	The vertebral-costal articulations posteriorly

Shoulder	The gleno-humeral joint, scapulothoracic articulation and acromioclavicualr joint

Chest	The manubrio-sternal joint, sternal-costal joint, costal-chondral joints and sternal-clavicular joint

Elbow	The ulnar-humeral articulation and the proximal radio-ulnar joint

Wrist	The radiocarpal joint, distal radio-ulnar joint and intercarpal joints

Hand	All joints distal to the wrist

* Soft tissue structures were defined as surrounding the involved joint as viewed from the anterior, medial, posterior and lateral aspect.

## Results

Over the course of the study a total of 487 treatment consultations were provided to the 29 intervention players (average of 16.8 treatment consultations per player), with all players being compliant to the minimum treatment protocol. This resulted in treatment being delivered to 2,000 joint based regions (47.0% total treatment) and 2,258 soft tissue based regions (53.0% of total treatment). On average per treatment consultation players received treatment to approximately 4 joint and 4 soft tissue based regions, which were not necessarily the same. Of the total treatment provided 65.3% was classified as being delivered to asymptomatic regions and 34.7% to symptomatic regions.

Figure 1 demonstrates the breakdown of joint based therapy into that for symptomatic and asymptomatic benefit. Of the total joint based therapy 73.5% was for asymptomatic benefit and 26.5% symptomatic benefit. The most common regions treated for asymptomatic benefit were the thoracic spine (21.3%), knee (20.5%), hip (19.0%), sacroiliac joint (12.5%) and lumbar spine (11.1%). The most common regions treated for symptomatic benefit were the lumbar spine (24.3%), thoracic spine (16.7%), hip (14.0%), cervical spine (13.3%), sacroiliac joint (10.8%) and knee (10.4%). Of interest the following ratios of asymptomatic: symptomatic treatment occurred at the knee (5.5:1), hip (3.8:1), thoracic spine (3.6:1), sacroiliac (3.2:1), and lumbar spine (1.3:1).

**Figure 1:** **Breakdown of joint based therapy into region and as being for symptomatic or asymptomatic benefit**.

Of the total joint based therapy delivered to the regions of the body, 55.7% was HVLA manipulation only, 35.9% a combination of HVLA manipulation and mobilization and 8.5% mobilization only. Therefore, 91.6% of the total joint based treatment involved some form of HVLA manipulation technique. When assessing the breakdown of HVLA manipulation techniques performed, 62.9% was manually performed and 37.1% mechanically assisted.

Figure 2 demonstrates the breakdown of soft tissue based therapy into that for symptomatic and asymptomatic benefit. Of the total soft tissue based therapy 58.0% was for asymptomatic benefit and 42.0% was for symptomatic benefit. The most common asymptomatic soft tissue regions treated were the gluteal region (22.0%), hip flexors (13.8%), knee (13.0%) and lumbar spine (10.6%). Only 5.6% of treatment was delivered to the posterior thigh. The most common soft tissue regions treated for symptomatic benefit were the gluteal region (21.5%), lumbar spine (14.2%), thoracic spine (7.6%) and posterior thigh (7.4%). Of interest the following ratios of asymptomatic: symptomatic treatment occurred at the knee (4.3:1), hip flexor (3.3:1), gluteal region (1.4:1) and lumbar spine (1.0:1).

**Figure 2:** **Breakdown of soft tissue based therapy into region and as being for symptomatic or asymptomatic benefit**.

## Discussion

This study documented that the sports chiropractic intervention applied in a recent RCT [21] comprised an ongoing, multi-region treatment approach incorporating both soft tissue techniques and joint based manipulation and mobilization. A number of joint and soft tissue structures were treated on each consultation, which were not necessarily the same. Whilst not being limited to manipulation only, there was an emphasis on HVLA manipulation techniques, with both manual and mechanically assisted techniques being performed, often in combination with mobilisation. A high proportion of treatment was provided to asymptomatic areas, particularly when joint based therapy was provided. With regards to joint based therapies delivered for asymptomatic benefit, treatment was predominantly delivered to the knee, hip, thoracic spine, sacroiliac joint and lumbar spine. For soft tissue therapies, asymptomatic treatment was predominantly delivered to the knee, hip flexor and gluteal region. When assessing ratios of asymptomatic and symptomatic treatment, the knee, hip and pelvic regions featured prominently for soft tissue and joint based therapies, which are all non-local to hamstring and lower-limb injury. No adverse events were associated with this treatment approach [21]. Based on the findings of the original RCT [21], the addition of this care experience appears to have improved the overall outcome for these players. However, it is important to note the preliminary nature of this research and the pragmatic nature of the study and that conclusions with respect to treatment effectiveness should be made with caution.

The sports chiropractic intervention was pragmatically and individually determined in a patient centered approach. In deciding what treatment to deliver and where to apply it, in particular for the large amount of asymptomatic treatment, several factors were considered. This included the patients current and previous medical history, particularly history of injury. This was combined with examination findings which included a postural assessment, observation of gait and motor patterns, static and motion palpation, range of motion assessment, various orthopaedic and other tests. The information gained from this was pooled together to make a clinical decision, such as occurs in clinical practice of all manual therapy professions. The multimodal and multi-region treatment approach delivered likely reflects the complex multi-factorial aetiology of hamstring and lower-limb injuries which have been said to result from a complex interaction of multiple risk factors and events, of which only a fraction have been identified [28]. In this regard, Dvorak et al. have highlighted the importance of multiple, simultaneous factors to develop a multidimensional predictor score for soccer injuries [29]. This could explain the reason for the amount of soft tissue and joint based treatment delivered on each treatment consultation, as an attempt was made to reduce all possible local and non-local risk factors for hamstring and lower-limb injury. The presence of multiple, simultaneous risk factors could highlight the importance of an effective multi-disciplinary environment providing a multimodal approach to injury prevention. Such an approach has been discussed as being necessary in hamstring injury management [30].

The use of joint based therapy in this study is of interest, as we contend that the biggest difference between the intervention and the best practice management applied to players (which included manipulative physiotherapy), was the addition of high amounts of HVLA chiropractic manipulation to a number of asymptomatic and symptomatic joint regions each treatment consultation. This study documented that 91.6% of joint based treatment involved HVLA manipulation and each treatment consultation involved manipulation or mobilisation to 4 regions. Although data was not included in this study on the management rendered by club staff, from the authors limited knowledge of the treatment provided in the control group, HVLA manipulation was rarely performed whilst the mechanically assisted techniques are exclusive to chiropractic. Previous research has shown that professions falling under the manual therapy banner do in fact have differing treatment methods [31]. Research investigating physiotherapist management of low back pain has shown that high-velocity spinal manipulation is used between 2.8% [32], 3.7% [33], 4.3% [34], 8.9% [35], and more recently in a heavily evidence based education system 36.2% of the time by a group of students [36], figures much lower than in this injury prevention RCT. Alternatively, low velocity mobilization is used between 27.2% [33], 43.8%[35], 58.6% [36], 58.9% [32], and 72% of the time [34]. More relevant to this study is research investigating sports physiotherapy scope of practice. Management provided by sports physiotherapists at international athletics competition has been shown to include asymptomatic treatment [16]. Published literature from the Olympic polyclinic has demonstrated that the most common modalities used are ultrasound (14.2% of total treatment), massage (13.5%), manual therapy techniques (13.4%), therapeutic exercise (12.4%), cryotherapy (9.3%), transcutaneous electrical nerve stimulation (TENS) (8.5%) and taping (7.9%) [18]. The use of manual therapies documented appears significantly lower than in this RCT. Similar literature from the Pan-American Games has also been performed [19]. The most common modalities used were kinesiotherapy (defined as muscle strengthening and/or flexibility exercises) (24.9% of all total treatments), ultrasound (19.4%), cryotherapy (17.2%), superficial heat (12.8%), interferential current (11.1%), TENS (7.3%), with osteopathy rarely used (0.6%) [19].

The findings of this study and the available literature suggest that the sports chiropractic intervention provided, in particular the amount, technique type and reason for HVLA manipulation is different to that of the clinical practice of physiotherapy. Although the management provided appeared to be reflective of published sports chiropractic and modern multimodal (MMM) chiropractic scope of practice [12-14], prospective clinical practice surveys of sports chiropractors do not exist. Such studies are encouraged which would allow assessment of the consistency between this research protocol and clinical practice and comparison with both physiotherapy and chiropractic clinical practice. As discussed by Hurley et al. [20], the results of this study should allow manual therapists to determine how closely the trial design, practitioner and interventions mimic their practice setting. Clinicians can then interpret and perhaps implement the evidence in a more meaningful way and the uptake of a similar treatment approach may have potential for injury prevention benefit as demonstrated in the RCT on a wider scale.

HVLA manipulative techniques are believed to return physiologic and accessory motion to hypomobile structures, correcting deficits in range of motion. Additionally short term strength changes in lower-limb musculature following spinal [37], and lower-limb [38] joint manipulative techniques have been observed. This may have contributed to improved hamstring and lower-limb muscle function and injury prevention in this study. It supports the hypothesis that hamstring and lower limb muscle strain involves a local and distant model [1,11,21]. Further indirect evidence for non-local factors having a role in injury causation exists in that a hamstring flexibility intervention in a military population has been shown to be capable of lowering the number of lower extremity overuse injuries [39], meaning improvements in knee injury in this RCT may have been a direct effect of treatment or through indirect improvements in hamstring function [21].

A large proportion of treatment was directed to the low back and pelvis. This is not surprising considering the incidence of low back injury and pain in Australian footballers [40]. The link between the low back and pelvis and hamstring and lower limb injuries has been discussed for some time [6,41]. Substantial treatment was also directed at the hip and knee. A large amount of treatment directed here was for the aim of asymptomatic or functional improvement. There has only been recent discussion on a possible link between these joints and hamstring and lower limb injury from the perspective of the kinematic chain [1,5,11]. The intricate anatomical attachments of the hamstring muscle to the knee [42], and fascial connections to the peroneus longus at the fibula [43], provide indirect evidence for knee and proximal tibial-fibular joint function to be of importance for hamstring function. This provides indirect support for the contention that non-local factors may play a role in hamstring and lower-limb injury causation [21].

Limitations exist in this study. Firstly, there are limitations in generalizing the results, as all treatment was provided by a single practitioner, who may not be representative of the chiropractic profession or the sports chiropractic subgroup of the profession. As the sports chiropractor in the study was working with the current best practice medical, paramedical and sports science team, it is highly likely that players would have consulted club medical or paramedical staff for treatment of symptomatic tissues, resulting in an under-reporting of symptomatic treatment, which may have occurred in clinical practice. When analysing the results of treatment rendered it should also be noted that some players consulted the sports chiropractor for management of injuries as they may have preferred the sports chiropractic approach for some conditions and because there is also a cultural phenomenon in many of the body contact sports that players do not want to be seen to be receiving treatment for injuries for fear of jeopardising team selection. Because the players were enrolled in an injury prevention study the stigma associated with treatment may have been lifted. Therefore it is not possible to say that all treatment may contribute to an injury prevention benefit, nor may results be entirely reflective of clinical sports chiropractic practice. As a multimodal treatment approach was applied in conjunction with a range of other therapies, it is also not possible to determine what resulted in the injury prevention. Further limitations of this study are that the results are likely biased towards asymptomatic treatment due to the injury prevention focus and again this may not accurately reflect clinical sports chiropractic practice.

The authors recommend this RCT be repeated in other sports with a high prevalence of hamstring and lower-limb injury. Future research would benefit from recording the nature of the control interventions in order to clarify the differences between interventions and to specifically address the role of HVLA based manipulative techniques. Additionally, the actual scope of practice of sports chiropractors needs to be documented and compared to the amount of treatment, the treatment techniques rendered, the location and frequency of treatment in this study to assess whether it is representative. This would allow for a multi-practitioner study to be conducted and allow more meaningful comparisons with both the physiotherapy and chiropractic professions.

## Conclusions

An individualized, ongoing multi-region and multimodal sports chiropractic intervention was applied in this cohort of semi-elite athletes. The sports chiropractic intervention aimed to reduce local and non-local risk factors to hamstring and lower limb muscle injury, although it can not be determined whether this occurred. A significant proportion of treatment was delivered to asymptomatic areas, particularly joint based therapies, which consisted largely of HVLA manipulation techniques, often in combination with mobilizations. However, the treatment was not limited to a manipulation only approach. Manual HVLA techniques were most commonly used although mechanically assisted techniques featured prominently. Publication of these findings allows manual therapists to determine how closely the trial design, practitioner and interventions mimic their practice setting. Clinicians not utilizing HVLA manipulation could consider higher utilization rates in a multimodal protocol over other more established interventions that have little to no evidence to support their use in the prevention of hamstring and other lower-limb injuries. However, it is important to note the preliminary nature of the evidence presented and the requisite for future studies to further explore this.

## Competing interests

The authors have no conflict of interest that is directly relevant to the content of this manuscript. No source of funding was used in the preparation of this manuscript.

## Authors' contributions

WH conceived the idea of the study with study design modified by HP. All treatment provided and recorded was by WH. WH and HP contributed to writing the multiple drafts and the final document. All authors read and approved the final manuscript.
